# IL-8 Is Upregulated in the Tissue-Derived EVs of Odontogenic Keratocysts

**DOI:** 10.1155/2022/9453270

**Published:** 2022-07-30

**Authors:** Jian-Feng Liu, Chen-Xi Zhang, Rui-Fang Li, Qi-Wen Man

**Affiliations:** ^1^The State Key Laboratory Breeding Base of Basic Science of Stomatology (Hubei-MOST) & Key Laboratory of Oral Biomedicine Ministry of Education, School & Hospital of Stomatology, Wuhan University, Wuhan, China; ^2^Department of Oral and Maxillofacial Head Neck Surgery, School & Hospital of Stomatology, Wuhan University, Wuhan, China

## Abstract

**Background:**

Interleukin 8 (IL-8) is a chemotactic cytokine released by various cells including leukocytes, endothelial cells, and epithelial cells. IL-8 has multiple functions in inflammation, tumour invasion, or angiogenesis. Human odontogenic cystic lesions are chronic and frequently inflamed. Tissue-derived extracellular vesicles (Ti-EVs) are widely present in various tissues and could more accurately reflect the characteristics of the primary tissue. However, the involvement of IL-8 in Ti-EVs of human odontogenic lesions is still unclear. This study aimed to explore the expression of IL-8 in Ti-EVs of human odontogenic lesions and the potential roles of Ti-EVs that carried IL-8.

**Methods:**

Fresh tissue samples of dentigerous cyst (DC, *n* = 5) and odontogenic keratocyst (OKC, *n* = 5) were collected for Ti-EVs isolation. Ti-EVs were characterised by transmission electron microscopy and nano-flow cytometry analysis. The cytokine profile of Ti-EVs was explored by cytokine antibody array. The IL-8 expression was examined by immunochemical staining in tissue of odontogenic lesions (DC, n =12; OKC, n =28). Antioxidants (N-acetyl-L-cysteine and diphenyleneiodonium) were employed to treat HaCaT cells, and the expression of IL-8 was detected by enzyme-linked immunosorbent assay. The gene expression of MMP9 was explored by quantitative real-time polymerase chain reaction in co-culture system of fibroblasts of OKC with Ti-EVs.

**Results:**

Compared with DC, the expression of IL-8 in Ti-EVs and fixed tissue specimens of OKC was markedly upregulated. The antioxidants decreased the expression level of IL-8 protein in the supernatant of HaCaT cells. The Ti-EVs treatment (10 *μ*g/ml) of fibroblasts significantly induced the MMP9 mRNA expressions in OKC fibroblasts.

**Conclusions:**

IL-8 was upregulated in Ti-EVs of OKC and might be involved in the tissue destruction of OKC.

## 1. Background

Odontogenic keratocysts (OKCs) are common jaw cysts, which were characterised by local invasiveness and high recurrence potential [1]. Genetic study revealed that a proportion of OKC lesions is related with a mutation or inactivation of the *PTCH1* gene [2]. The bacterial products are commonly present in the jaw cystic lesions; thus, various cytokines and chemokines are widely distributed in the microenvironment of the odontogenic lesions [3]. In addition, during the progression of OKCs, degradation of supporting tissues and jaw bone can be observed accompanied by the alternative expression of cytokines, matrix metalloproteinases (MMPs), interleukins (ILs), and chemokines [4]. Accumulating studies showed the crucial roles of MMPs in regulating homeostasis, degradation, and reconstruction of the extracellular matrix (ECM) in pathologic and physiological conditions [4, 5]. The aberrant level of the cytokines or chemokines could break the balance between the homeostasis of the immune microenvironment and bone metabolism. However, the regulatory roles of cytokines in the enlargement of OKCs are still unexplored.

Extracellular vesicles (EVs) are lipid-bilayer membrane structures secreted by most cell types [6]. EVs act as messengers via the horizontal transfer of lipids, proteins, and nucleic acids; they influence various pathophysiological processes in parent and recipient cells [6]. Previous studies focused on the cell-line derived or body fluid-derived EVs, which were relatively easy to isolate [6–8]. However, the cell-line derived EVs are not representative of the disease study, and the body fluid-derived EVs are enriched in the contaminations, such as immunoglobulins and blood cell-derived substances [9]. Compared with the body fluid-derived EVs or cell line-derived EVs, tissue-derived EVs had the advantage of tissue specificity and accurate reflection of tissue microenvironment [9]. However, the tissue-derived EVs had not been illuminated in odontogenic tissues. Cytokines are soluble proteins that mediate cell–cell communication in the body [10]. Cytokines are generally thought to be released and functioned as soluble molecules [10]. However, we found that bioactive cytokines, especially specific cytokines, could be packaged into the EVs. In addition, the cytokine profile of the tissue-derived EVs in odontogenic cysts remains unknown.

Interleukin-8 (IL-8) is a chemoattractant cytokine produced by various cells including leukocytes, endothelial cells, and epithelial cells [11]. Report showed that endothelial cells store IL-8 in their storage vesicles named the Weibel–Palade bodies [12]. Originally, IL-8 was identified as neutrophil chemoattractant via binding to the receptors CXCR1/2 [13]. In addition, IL-8 was reported to promote integrin *β*3 upregulation and the invasion of hepatocellular carcinoma cells through activation of the PI3K/Akt pathway [14]. Oral cavity hosts a bacterial environment, which was related with physiological barrier, caries, and bad oral breath habit [15]. In odontogenic lesions, IL-8 had been proven to be highly expressed in ameloblastoma epithelial cells and irreversible pulpitis [16, 17]. We isolated Ti-EVs of odontogenic lesions and compared the cytokine profiles from DC and OKC patients. We showed that IL-8 was predominantly enriched in OKC Ti-EVs, and the level of IL-8 was closely related with reactive oxygen species (ROS) production. This study initially investigated the cytokine profile of Ti-EVs of odontogenic lesions and implied that Ti-EVs containing IL-8 might be related with the progression of OKC, which might be a potential target for OKC treatment.

## 2. Materials and Methods

### 2.1. Single-Cell Suspension from OKC and DC Tissue

The tissue samples of odontogenic keratocyst (OKC) and dentigerous cyst (DC) were collected from the Department of Oral and Maxillofacial Surgery, School and Hospital of Stomatology, Wuhan University. The tissue was rinsed with phosphate-buffered saline (PBS) in an effort to remove blood clots and impurities. The weight of the collected tissue was measured using milligram balance. The tissue samples were gently washed twice by PBS and cut into pieces (~2 × 2 × 2 mm) using scissors. Enzymes are used at the following concentrations: collagenase D (1 mg/ml, Sigma-Aldrich, Germany) and DNase I (40 U/ml, Sigma-Aldrich, Germany). Based on the weight of the tissue, the appropriate volume of enzymes was thawed. This step allows EVs to be released from the tissue, where they are entrapped. Then, the mixture was placed at 37°C for 1 hour in the mechanical horizontal rotators. A 0.70 *μ*m pore size filter was applied to remove the largest elements among the suspension.

### 2.2. Ti-EVs Isolation

The supernatant was centrifuged at 10,000 × *g* for 30 min to remove large vesicles using the Centrifuge 5810R (Eppendorf, Germany), followed by ultracentrifugation at 120,000 × *g* for 70 min (Optima XE, Beckman Coulter, USA). The Ti-EVs pellet were resuspended in 100 *μ*l of Phosphate-Buffered Saline (PBS, Gibco, USA) and ultracentrifuged at 120,000 × *g* for 70 min and transferred to Eppendorf tubes. The collected Ti-EVs were stored at −80°C for further examination.

### 2.3. Transmission Electron Microscopy (TEM)

TEM was performed at the Servicebio, Wuhan, China. Ti-EVs were mounted onto copper-coated TEM grids for detection. The grids were stained with 1% *v*/*v* uranyl acetate, and the Ti-EVs were captured using the Hitachi HT7700 transmission electron microscope (Hitachi, Ltd., Tokyo, Japan).

### 2.4. Nano-flow Cytometry

An amount of 1 *μ*l antibodies was incubated with 10 *μ*l Ti-EVs. The following antibodies were used: PE-conjugated CD63 (1 : 10, 353003; BioLegend). Samples were incubated with the above antibodies at 4°C for 1 hour. Data were collected with an A60-Micro Plus nanoscale flow cytometer (Apogee Flow Systems Inc., Northwood, UK) and analysed using FlowJo software (VX.0.7) for nano-flow cytometry analysis.

### 2.5. Cytokine Antibody Array

For cytokine antibody array, equal quality of Ti-EVs (50 *μ*g protein, DC- and OKC-derived Ti-EVs) were loaded for analysis. Following the manufacturer's protocols, cytokines and chemokines were detected using Bio-Plex Pro Human Cytokine Screening 40-plex Panel using Bio-Plex MAGPIX System (Bio-Rad) (Wayen Biotechnologies (Shanghai), Inc.).

### 2.6. Enzyme-linked Immunosorbent Assay (ELISA)

Standard IL-8 proteins were prepared using Human Interleukin 8 (IL-8) ELISA Kit (CUSABIO, Wuhan, China). Standard IL-8 protein (2000, 1000, 500, 250, 125, 62.5, and 0 pg/ml) or Ti-EV samples of 100 *μ*l (50 *μ*g) were added to each well, mixed gently, and incubated at 37°C for 1 hour. After the liquid is removed, 100 *μ*l of biotin-antibody (1x) was added to each well and incubated for 1 hour at 37°C. Then, the liquid was discarded and washed by 200 *μ*l washing solution per well. Horseradish peroxidase (HRP)-Avidin (1x) working solution 100 *μ*l was added to each well and incubated at 37°C for 1 hour. After washing, 90 *μ*l of substrate solution was added to each well in sequence, and color was developed at 37°C for 15–30 minutes away from light. Finally, 50 *μ*l stop solution was added to each well in sequence to stop the reaction. Within 5 minutes after the termination of the reaction, the optical density (OD) of each well was measured in sequence at 450 nm with a microplate reader (Bio-Tek, USA).

### 2.7. Cell Treatments

HaCaT cells were seeded at a starting density of 1 × 10^5^ cells/dish in growth medium (DMEM with high glucose, Hyclone) supplemented with 10% FBS in 6 cm dishes. The cells were then allowed to adhere to the wells in the incubator prior to treatments. Cells, which were typically ~80%–90% confluent, were treated with 1 mM NAC (the scavenger of ROS, Beyotime, China) or 10 *μ*M diphenyleneiodonium chloride (ROS inhibitor, Beyotime, China) for 6 hours. Controls and the treated supernatant samples were collected and tested for IL-8 levels. In addition, HaCaT cells were treated with thapsigargin (2 *μ*M, Selleck, USA) or the NF-*κ*B inhibitor (BAY 11-7082, 2 *μ*M, Selleck, USA). Thapsigargin is a noncompetitive inhibitor of the sarco/endoplasmic reticulum Ca^2+^ ATPase, which could raise cytosolic (intracellular) calcium concentration by blocking the ability of the cell to pump calcium into the sarcoplasmic and endoplasmic reticula.

### 2.8. [Ca^2+^] Measurement Assay

The intracellular Ca^2+^ concentration in the cyst fluid or supernatant of HaCaT cells was detected by a calcium colorimetric assay kit (Beyotime, China). The HaCaT cells (control group and thapsigargin treated group) were lysed with lysate buffer. Then, 50 *μ*l chromogenic reagent and 50 *μ*l calcium assay buffer were added to the 50 *μ*l cell lysates, followed by the 5 min incubation. Finally, the incubation buffer was loaded in the 96-well microplate reader (Bio-Tek, USA) and then measured with the absorbance at 575 nm.

### 2.9. Intracellular ROS Level Detection by Dihydroethidium

The intracellular ROS levels of HaCaT cells were assayed using the fluorescence probe dihydroethidium (DHE, Beyotime, China). The HaCaT cells were cultured in slides and treated with the fluorescence probe dihydroethidium. The fluorescence image of the stained cells in the suspension was immediately photographed using fluorescence microscope. The mean intensity of DHE-stained HaCaT cells was calculated by ImageJ 1.52 software.

### 2.10. Primary Fibroblast Culture and Treatment

The primary fibroblast of odontogenic keratocyst was cultured with tissue culture method. Odontogenic keratocyst tissue was cut into 5∗5 mm cubes. The cubes were placed on the culture disk for 2 h in an incubator with 5% CO_2_ at 37°C humidified atmosphere. Then, culture medium (DMEM, Hyclone+10%FBS, CellMax, China) was added to the culture disk. The culture medium was replaced every three days. At day 7, the spindle-shaped cells were grown in the surroundings of tissue cubes. The Ti-EVs were filtrated with a Millex-GV Filter (0.22 *μ*m, Merck Millipore, USA). After filtration, Ti-EVs (10 *μ*g/ml) were cocultured with fibroblasts or IL-8 neutralisation (Genetex, 10 *μ*g/ml, 2 h, USA) treated fibroblasts.

### 2.11. Phalloidin Staining of OKC Fibroblast

The original medium was abandoned, and the cells were washed twice with PBS. After the cells were fixed with 4% formaldehyde solution at room temperature, the cells were cleaned with PBS two to three times for 10 min each. Cells were permeated with 0.1%–0.5% Triton X-100 solution for 5 min. The permeating solution was removed and washed with PBS two to three times for 10 min each. The working solution of phalloidin (Abcam, ab235138, UK) was added to cover the cells, and the cells were incubated for 30 min at room temperature away from light. The cells were cleaned three times with PBS for 5 min each. The nuclei were restained according to the DAPI (4',6-diamidino-2-phenylindole) staining solution instructions. The image of the stained cells was immediately photographed using fluorescence microscope.

### 2.12. Immunohistochemistry Staining

The tissue microarray (TMA) of odontogenic lesions including 11 cases of DC and 30 cases OKC was constructed by Servicebio, Wuhan, China. The TMA of odontogenic lesions was incubated in 65°C for 2 h. The slides of TMA were dewaxed by xylene and dehydrated by graded ethanol. For antigen exposure, the slides were boiled in the electric pressure cooker and cooked to 120°C for 60 seconds. After cooling to the room temperature, the slides were blocked by goat serum. The primary antibody IL-8 (1 : 200, Proteintech, China) was incubated with the slides overnight and followed by HRP-conjugated solutions. Finally, the slides were stained with diaminobenzidine (Zhongshan Golden Bridge Biotechnology Co. Ltd., China) and hematoxylin staining solution (Servicebio, Wuhan, China).

### 2.13. Immunohistochemical Scoring

The slides of odontogenic lesions were scanned and photographed by a digital pathological slice scanner (3DHISTECH Pannoramic MIDI, Hungary). Aperio Image Scope CS2 scanner (CA, USA) was used for tissue slide scan. Aperio Quantification software (Version 9.1) was applied for the quantification. The epithelial area of the tissue was manually selected for quantification. Then, the formula (1 × the percentage of weakly positive staining) + (2 × the percentage of moderately positive staining) + (3 × the percentage of strongly positive staining) was used for the analysis of the staining scores. The scaled values (*H*-scores) of IL-8 expressions were subsequently converted to the dataset for analysis.

### 2.14. EVs Uptake Assay

The Ti-EVs were incubated with carboxyfluorescein succinimidyl ester (CFSE, Thermo Fisher, 2 *μ*m) for 20 min under 37°C. The fibroblasts were stained with Dil solution (5 *μ*M, 10 min, Thermo Fisher, D3911, USA). The CFSE-labelled Ti-EVs were cocultured with Dil-stained fibroblasts for 2 h. Then, the supernatant was removed and washed by PBS. The fibroblasts were photographed using a fluorescence microscope (Beckman Coulter, USA).

### 2.15. Real-Time Quantitative Polymerase Chain Reaction (RT-qPCR)

Total RNA was isolated from OKC fibroblasts (control group, Ti-EVs co-cultured group and IL-8 neutralisation (Genetex, 10 *μ*g/ml, USA) plus Ti-EVs cocultured) using TRIzol reagent (Invitrogen, USA), according to manufacturer's instructions. cDNA was made from total RNA using reverse transcriptase kit (TaKaRa Shuzo, Kyoto, Japan), which was amplified on an Applied Biosystems 7500 real-time PCR system (Foster City, CA, USA). The specific primers (Invitrogen, USA) for MMP9 were 5′-TGTACCGCTATGGTTACACTCG-3′ (forward) and 5′-GGCAGGGACAGTTGCTTCT-3′ (reverse). The specific primers for GAPDH were 5′-GGAGCGAGATCCCTCCAAAAT-3′ (forward) and 5′-GGCTGTTGTCATACTTCTCATGG-3′ (reverse). The thermal cycling conditions comprised 94°C for 30 sec, 60°C for 1 min, 72°C for 1 min, and a final elongation at 72°C for 10 min, amplifying for 38 cycles. The 2^−*ΔΔ*CT^ method was used for data analysis.

### 2.16. Statistics

Statistical analyses were performed with Prism 7.0 software (GraphPad). All results were presented as mean ± SD. Differences of data between two groups were assessed by Mann–Whitney test; one-way ANOVA test or Brown-Forsythe and Welch ANOVA test was used when the data met the normal distribution, and use the Kruskal-Wallis test for data that did not meet the normal distribution. *P* value < 0.05 was considered statistically significant.

## 3. Results

### 3.1. Characterisation of Tissue-Derived EVs of DC and OKC

To isolate the tissue-derived EVs, mechanical slicing and collagenase were used to free the EVs within tissue interstitial space. After ultracentrifugation, the tissue-derived EVs were collected and stored. Transmission electron microscopy was performed to explore the characteristics of tissue-derived EVs, and the results showed that membrane vesicles ranging about 100 nm were observed (Figure 1(a)). Nano-flow cytometry was employed to further quantify the CD63 expressions in the surface of tissue-derived EVs, and the results showed that about 30% of tissue-derived EVs were positive for CD63 in the surface (Figure 1(b)).

### 3.2. IL-8 Was Highly Expressed in Tissue-Derived EVs and Fixed Tissue Specimens of OKC

A total of 50 *μ*g proteins of Ti-EVs were loaded by cytokine antibody array for the cytokine antibody array. Among the 27 types of cytokines tested, IL-8, RANTES, and FGF were at high concentrations (Figure 1(c)). Ti-EVs from OKC samples (*n* = 5) showed significantly higher level of IL-8 than the Ti-EVs of DCs (*n* = 5) (Figure 1(d)). To explore the IL-8 expression in tissues, tissue microarray, including DCs and OKCs, was employed for IL-8 evaluation. The results also showed that IL-8 was slightly upregulated in the epithelial cells of OKC (*n* = 28) compared with DC (*n* = 12) (Figures 2(a) and 2(b)).

We collected the cyst fluid of OKC and tested for the Ca^2+^ concentration to evaluate the Ca^2+^ concentration within cyst fluid. The result showed that the Ca^2+^ concentration of cyst fluid of OKC was about 1.2 mmol/l (Figure 2(c)). In HaCaT cells, TG (thapsigargin, 2 *μ*M) treatment significantly upregulated the Ca^2+^ concentration in 90 s (Figure 2(d), *P* < 0.05). In addition, the TG treatment (2 *μ*M, 3 h or 6 h) also induced the elevated IL-8 expressions within the supernatant of HaCaT cells in 6 h (Figure 2(d)). In addition, the NF-*κ*B inhibitor (BAY 11-7082) was used to test the potential role of the NF-*κ*B signalling pathway in TG-treated HaCaT cells (Figure 2(e)). The result showed that NF-*κ*B signalling pathway inhibition could lower the IL-8 levels of HaCaT cells although without significance. Higher intracellular level of Ca^2+^ could lead to the ROS production and NF-*κ*B signalling pathway activation. We also evaluated the intracellular ROS levels after TG treatment. We found that after 2 h of treatment with TG, the intracellular ROS was significantly unregulated by H_2_O_2_ probe (dihydroethidium) (Figures 3(a) and 3(b), *P* < 0.01). We also tested two antioxidants for IL-8 expressions. The result showed that adding antioxidants (N-acetyl-L-cysteine, diphenyleneiodonium) could significantly decrease the IL-8 protein level within the supernatant of HaCaT cells (Figure 3(c), *P* < 0.01 and *P* < 0.001, respectively).

### 3.3. EVs Containing IL-8 Promote MMP9 Expressions in OKC Fibroblasts

To further evaluate the biological effects of Ti-EVs, primary fibroblasts were cultured from fresh tissue of OKC. The phalloidin staining showed that OKC fibroblasts showed spindle-shaped cells (Figure 4(a)). The EVs uptake assay also revealed that CFSE-labelled EVs could be uptaken by OKC fibroblasts within 2 h (Figure 4(b)). The OKC fibroblasts were cocultured with Ti-EVs, and the mRNA level of MMP9 was determined by RT-qPCR. The results showed that the mRNA level of MMP9 was significantly upregulated after Ti-EVs treatment for 12 h; it was partially blocked by IL-8 neutralising antibody without significance (Figure 4(c)). This result showed that Ti-EVs carrying IL-8 could induce the MMP9 mRNA upregulation in OKC fibroblasts.

## 4. Discussion

The findings of this study clearly showed that IL-8 was enriched in Ti-EVs of OKC compared with the cytokines of Ti-EVs of DC. In addition, the calcium influx significantly elevated the ROS level of HaCaT cells and induced the IL-8 levels within the supernatant of cultured epithelial cells. The Ti-EVs of OKC significantly upregulated the mRNA level of MMP9 in OKC fibroblasts. These results initially showed the cytokine profile of Ti-EVs of OKC and implied the potential role of Ti-EVs for supporting bone resorption.

Tissue-derived EVs have several characteristics compared with cell-line derived or body fluid-derived EVs [9, 18]. EVs in body fluids are heterogeneous, originating from different cellular origins and from diverse sources [19, 20]. Tissue-derived EVs could reflect the characteristics of specific tissues and lowered the contamination of plasma proteins or immune globulin, which were widely present in the serum or saliva [18, 19]. Until now, no studies revealed the cytokine profiling of tissue-derived EVs in odontogenic lesions. Herein, we employed the enzyme digestion method to isolate the tissue-derived EVs and analysed the cytokine profile of odontogenic lesions.

IL-8 had been previously determined in odontogenic lesions [16, 17, 21, 22]. Compared with healthy dental pulps, inflamed pulps present higher amounts of IL-1*β* and IL-8 [17]. In ameloblastoma, coculture of ameloblastoma cells and bone marrow stromal cells significantly upregulate the expression of IL-8, which was related with the bone resorption of ameloblastoma [16]. Using tissue culture model, the IL-8 was detected in radicular cyst and odontogenic keratocyst [21]. In the test of aspirate from jaw cysts, the study also found a significant elevation of IL-8 in OKC compared with ameloblastoma and dentigerous cyst (*P* = 0.028) [22]. In the present study, we use immunohistochemistry staining method, showing that IL-8 was mainly expressed in the epithelium of odontogenic lesions. This finding implies that the epithelial cells might be the main cellular origins of IL-8.

Calcium is a vital mineral, which is crucial for hard tooth enamel formation and bone health [23]. In the serum, the concentration of free ionised calcium was 1.15 mmol/l to 1.29 mmol/l [24]. Similar to the serum-ionised calcium levels, the cyst fluid level of ionised calcium (~1.2 mmol/l) was similar to the level of serum-ionised calcium levels. This finding was in accordance with fluid exchange between cyst fluid and serum. The tissue transient calcium level of odontogenic cysts is still unexplored due to the lack of animal model and instantaneous detection of calcium. The bone resorption process might result in the liberation of calcium and other mineral elements. However, in jaw cyst lesions, the bone resorption rate is very low to induce the significant elevations of calcium in the cyst fluid or tissue. In addition, several pathways can lower the calcium levels including urinary excretion or regulation by calcium sensing receptors.

ROS is the by-product of oxygen metabolism, and ROS plays vital roles in various diseases [25]. As a host defence mechanism against bacterial pathogens, the generation of ROS performed by NADPH oxidase is essential in phagocytic infiltration-related diseases [25, 26]. A study demonstrated that thapsigargin (TG) induces depletion of Ca^2+^ stores, elevating [Ca^2+^]i [27]. In this study, we employed TG to induce the calcium influx and the ROS levels. Odontogenic cystic lesions are frequently inflamed and induced by the bacterial pathogens. A high concentration of ROS and long-term exposure to ROS could lead to cellular damage [26, 28]. Nuclear factor *κ*-light-chain-enhancer of activated B cell (NF-*κ*B) activation and cellular death are important mechanisms of ROS-mediated exacerbating inflammation [29]. A previous study illustrated that iNOS was overexpressed in OKCs when compared with DCs and radicular cyst, suggesting that iNOS may contribute to the aggressive behaviour of OKC [30]. This finding showed that ROS may play vital roles in inflammatory and developmental cyst lesions. In periapical granulomas, iNOS-positive cells might play a critical role in the activation of macrophages through the induction of NO and might modulate the degree of inflammation [31]. In apical periodontitis, positive correlation of the levels of IL-8 and NO suggests an involvement of neutrophil-derived NO in the pathogenesis of apical periodontitis [21]. In A549 cells, treatment of A549 cells with antioxidants decreased ROS production and expression of IL-8 mRNA [32]. Under hypoxic condition, normal human nasal epithelium cells could translocate HMGB1 into the extracellular area, depending on ROS production and involved in the upregulation of IL-8 [33]. Similar to a previous study, we found that antioxidants (ROS inhibitors) could significantly decrease the IL-8 levels within supernatant of HaCaT cells.

In tumour tissue, tumour-associated fibroblasts play a crucial role in tumour microenvironment and are also the most important cell type [34]. In odontogenic keratocysts, fibroblasts are also the dominant cell type in many characteristics similar to those of tumours, leading to the absorption and regeneration of bone tissue [35]. Tumour cells and fibroblasts communicate with each other, including autocrine and paracrine factors, including IL-8, resulting in the upregulation of MMP2 and MMP9 degradable extracellular matrix (ECM) components that trigger tumour invasion [36]. In trophoblast cell, the study also revealed that IL-8 could bind to CXCR1 and CXCR2, resulting in higher level of MMPs and integrins [37]. However, Ti-EVs stimulated fibroblasts showed significantly higher elevation of MMP9 (about four folds) than the results of trophoblast cell. The combined effects of various cytokines (RANTES, FGF, and MCP-1) and unexplored proteins might explain the remarkable elevations of MMP9.

However, this study has some limitations. Firstly, although EVs containing IL-8 have biological effects, whether the IL-8 was located in the surface or the inside of EVs is still unexplored. Second, a relatively small sample size was employed to confirm the IL-8 expressions in the Ti-EVs of OKC and DC.

In conclusion, we initially isolated tissue-derived EVs of odontogenic cystic lesions, mapped the cytokine profile of OKC, and explored the regulatory role of ROS in IL-8 production.

## Figures and Tables

**Figure 1:** Cytokine profile of tissue-derived EVs of odontogenic lesions. (a) Transmission electron microscope of collected odontogenic cyst-derived EVs. (b) Nano-flow cytometry analysis of EV marker (CD63) in collected odontogenic cyst-derived EVs. (c) Cytokine array analysis of collected odontogenic cyst-derived EVs. (d) Statistical analysis of IL-8 and RANTES levels in dentigerous cyst- and odontogenic keratocyst-derived EVs.

**Figure 2:** IL-8 expression in tissues of odontogenic lesions and IL-8 secretion is regulated by the NF-*κ*B signaling pathway in HaCaT cells. (a, b) Representative immunohistochemical staining and score of IL-8 in odontogenic lesions including dentigerous cyst (*n* = 12) and odontogenic keratocyst (*n* = 28). (c) The calcium level within the cyst fluid of odontogenic keratocyst (*n* = 3) was calculated. (d) Thapsigargin (2 *μ*M) significantly upregulated the intracellular calcium level within HaCaT cells in 90 seconds. (e) Thapsigargin significantly upregulated the protein level of IL-8 in HaCaT cells and partially reduced by NF-*κ*B inhibitor (BAY 11-7082, 2 *μ*M) in 6 h.

**Figure 3:** Stimulation of HaCaT cells with thapsigargin induces ROS production and IL-8 secretion. (a) Immunofluorescent staining of ROS level of HaCaT cells after thapsigargin treatment (scale bar = 10 *μ*m). (b) Thapsigargin significantly elevated the ROS level of HaCaT cells (thapsigargin 2 *μ*M, 6 h). (c) ROS inhibitors including N-acetyl-L-cysteine (2 *μ*M, 6 h) and diphenyleneiodonium (10 *μ*M, 6 h) significantly lowered the IL-8 expressions in HaCaT cells.

**Figure 4:** OKC tissue-derived EVs could elevate OKC fibroblast MMP9 expression via IL-8. (a) Representative image of cytoskeleton staining of OKC fibroblasts (scale bar = 10 *μ*m). (b) Representative image of tissue-derived EVs uptake by OKC fibroblasts (scale bar = 10 *μ*m). (c) The relative mRNA level of MMP9 in tissue-derived EVs cocultured and IL-8 neutralisation-treated OKC fibroblasts.

## Data Availability

All data generated or analysed during this study are included in this published article.
